RETRACTED

# Long non-coding RNA ANRIL alleviates H_2_O_2_-induced injury by up-regulating microRNA-21 in human lens epithelial cells

**DOI:** 10.18632/aging.102800

**Published:** 2020-04-20

**Authors:** Shanshan Du, Jingzhi Shao, Ying Qi, Xuhui Liu, Jingjing Liu, Fengyan Zhang

**Affiliations:** 1 Department of Ophthalmology, The First Affiliated Hospital of Zhengzhou University, Zhengzhou 450052, Henan, China

**Keywords:** cataract, H_2_O_2_, human lens epithelial cells, lncRNA ANRIL, microRNA-21

## Abstract

The accurate role of ANRIL in cataract is poorly understood. We aimed to reveal the effects of ANRIL on H_2_O_2_-treated HLECs, SRA01/04, as well as the regulatory mechanisms. Oxidative stress model of HLECs was induced by H_2_O_2_. Cell injury was evaluated according to cell proliferation, apoptosis and DNA damage using CCK-8 assay/flow cytometry and TUNEL assays/γH2AX staining. Expressions of ANRIL and miR-21 in HLECs were determined by RT-qPCR. The effects of miR-21, miR-34a and miR-122-5p inhibition as well as AMPK and β-catenin on HLECs with ANRIL overexpression and H_2_O_2_ stimulation were analyzed. *In vivo* experiment was performed via RT-qPCR. H_2_O_2_ repressed proliferation and induced apoptosis or DNA damage in HLECs. Those alterations induced by H_2_O_2_ were attenuated by ANRIL overexpression. MiR-21 was positively regulated by ANRIL, and both of them were repressed in H_2_O_2_-induced HLECs and cataract patient tissues. Inhibition of miR-21 but not miR-34a or miR-122-5p reversed the effects of ANRIL on H_2_O_2_-treated HLECs. Phosphorylation of AMPK and expression of β-catenin were increased by ANRIL via regulating miR-21. AMPK and β-catenin affected beneficial function of ANRIL-miR-21 axis.

Therefore, lncRNA ANRIL attenuated H_2_O_2_-induced cell injury in HELCs via up-regulating miR-21 via the activation of AMPK and β-catenin.

## INTRODUCTION

Cataract is the loss of normal transparency of the crystalline lens, which can reduce light transmission to the retina, resulting in decreased visual acuity and functional disability [1, 2]. As a leading cause of blindness, cataract accounts for approximately half of the cases of blindness worldwide [3]. As estimated, the number of people suffered cataract in the United States is going to reach 50 million by the 2050 due to the increase of life expectancy [4]. Currently, several risk factors such as diarrhea, aging, sunlight, smoking, diabetes, malnutrition, hypertension and renal failure have been identified for cataract formation [5, 6]. Previous studies have proved that the apoptosis of lens epithelial cells is a common cellular basis for the formation of non-congenital cataract in human and mammalians [7, 8]. Therefore, proliferation and apoptosis of lens epithelial cells are of great importance for development of cataract.

RETRACTED

Long non-coding RNAs (lncRNAs) are transcripts greater than 200 nucleotides without protein-coding potential [9]. Recently, an increasing number of lncRNAs have been identified to participate in cataract development, such as lncRNA TUG1 [10] and lncRNA MIAT [11]. Antisense non-coding RNA in the INK4 locus (ANRIL), also known as CDKN2B-AS, is a 3.8 kb lncRNA transcribed in the antisense direction of the *INK4B*-*ARF*-*INK4A* gene cluster [12]. Genome-wide association studies have shown that ANRIL is a genetic susceptibility locus shared associated by coronary disease, intracranial aneurysm and also type 2 diabetes [13]. Cataract is one of the most frequently observed complications of diabetes [14], and a meta-analysis involving 20837 subjects has illustrated that type 2 diabetes is a risk factor of cataract [15]. Hence, there might be a correlation between lncRNA ANRIL and cataract. However, the functional role of lncRNA ANRIL in cataract is poorly understood.

There are high concentrations of crystalline proteins in lens fibres, contributing to lens transparency and refractive properties [16]. Aggregation of crystalline proteins is the single most important factor in the development of cataract [17]. Despite mutation of crystalline proteins, oxidative stress may induce oxidative damage to the crystalline proteins, resulting in protein-protein disulfide formation and protein aggregation [18]. Previous studies have found that H_2_O_2_ can induce epithelial cell damage and protein degradation, which is followed by cataract formation [19, 20]. Therefore, human lens epithelial cells (HLECs) under stimulation with H_2_O_2_ were used to mimic cataract. In the present study, the SV40 T-antigen-transformed human lens epithelial cell line, SRA01/04, was used. Effects of lncRNA ANRIL on H_2_O_2_-induced cell injury were explored for the first time. Moreover, we also studied the possible downstream factor of lncRNA ANRIL as well as the involved kinases.

## RESULTS

### H_2_O_2_ induced HLEC injury

In order to examine the effects of H_2_O_2_ on HLEC, we performed this experiment. After stimulation with 400 μM H_2_O_2_, cell viability, expression of p53, cyclinD1 and CDK4, apoptosis and expression of proteins related to apoptosis in HLEC SRA01/04 cells were all measured. In Figure 1A, 1B, viability of cells was stimulated with different concentrations of H_2_O_2_ and viability under the 200, 300, 400, 500 and 600 μM H_2_O_2_ was significantly lower than that of the non-treated cells (*P* < 0.05, *P* < 0.01 or *P* < 0.001). The 400 μM was used in the following experiments. Compared with the control group, p53 protein expression was remarkably up-regulated (*P* < 0.001) whereas expression of cyclinD1 and CDK4 was markedly down-regulated (*P* < 0.05) after H_2_O_2_ stimulation (Figure 1C, 1D). In the meantime, percentage of apoptotic cells in the H_2_O_2_ group was dramatically higher than that in the control group (*P* < 0.001, Figure 1E, 1F). Consistently, H_2_O_2_ induced up-regulated Bax and cleaved caspase-3 as well as down-regulated Bcl-2 (Figure 1G). The γH2AX staining positive cells were increased by H_2_O_2_ induction (*P* < 0.001, Figure 1H). Results talked above indicated that H_2_O_2_ induced cell injury in HLECs.

RETRACTED

**Figure 1:** **H_2_O_2_ induced HLEC injury. HLEC SRA01/04 cells were treated with 400 μM H_2_O_2_ for 1 h, and non-treated cells were acted as control.** (**A**, **B**) Cell viability was measured by CCK-8 assay. (**C**, **D**) Expression of p53, cyclinD1 and CDK4 was testified by Western blot analysis. (**E**, **F**) Percentage of apoptotic cells was quantified by flow cytometry assay and TUNEL assay. (**G**) Expression of proteins related to apoptosis was detected by Western blot analysis. (**H**) γH2AX staining for detection of DNA levels. Data are shown as the mean ± SD of three independent experiments. *, *P* < 0.05; **, *P* < 0.01; ***, *P* < 0.001.

### Overexpression of lncRNA ANRIL attenuated H_2_O_2_-induced HLEC injury

For exploring the function of lncRNA ANRIL in H_2_O_2_-induced HLEC injury, the transfection experiment was performed. Recombined plasmid and empty pcDNA3.1 were respectively transfected into HLEC SRA01/04 cells, and expression of lncRNA ANRIL was determined. In Figure 2A, the expression level of lncRNA ANRIL in cells transfected with pc-ANRIL was observably higher than that in cells transfected with pcDNA3.1 (*P* < 0.01), suggesting that lncRNA ANRIL was overexpressed successfully after cell transfection. Then, transfected or untransfected HLEC SRA01/04 cells were treated with H_2_O_2_, and cell injury was evaluated. Results showed that H_2_O_2_-induced cell injury was alleviated by overexpression of lncRNA ANRIL, presenting increased cell viability (*P* < 0.05, Figure 2B), down-regulated p53 as well as up-regulated cyclinD1 and CDK4 (all *P* < 0.05, Figure 2C, 2D), also the decreased apoptotic cells (*P* < 0.05, Figure 2E, 2F), and down-regulated Bax and cleaved caspase-3 as well as up-regulated Bcl-2 (Figure 2G), when compared to the H_2_O_2_ + pcDNA3.1 group. But, the γH2AX staining positive cells were decreased by lncRNA ANRIL overexpression (*P* < 0.05, Figure 2H). Also, we detected that only p15 was affected, the protein expression levels of p14 and p19 were not influenced at all (Figure 2I). Results indicated that lncRNA ANRIL might attenuate H_2_O_2_-induced cell injury in HLECs.

RETRACTED

**Figure 2:** **LncRNA ANRIL attenuated H_2_O_2_-induced HLEC injury.** HLEC SRA01/04 cells were transfected with pcDNA3.1 or pc-ANRIL, and untransfected cells were acted as control. (**A**) Expression of lncRNA ANRIL was determined by RT-qPCR. Transfected or untransfected SRA01/04 cells were treated with 400 μM H_2_O_2_ for 1 h, and non-treated cells were acted as control. (**B**) Cell viability was measured by CCK-8 assay. (**C**, **D**) Expression of p53, cyclinD1 and CDK4 was testified by Western blot analysis. (**E**, **F**) Percentage of apoptotic cells was quantified by flow cytometry assay. (**G**) Expression of proteins related to apoptosis and (**I**) p14, p15 and p19 were detected by Western blot analysis. (**H**) γH2AX staining for detection of DNA levels. Data are shown as the mean ± SD of three independent experiments. *, *P* < 0.05; ***, *P* < 0.001.

### Overexpression of lncRNA ANRIL up-regulated miR-21 expression

To examine the regulation between the ANRIL and miR-21, the correlation between lncRNA ANRIL expression and miR-21 expression was subsequently explored. In Figure 3, miR-21 level in cells overexpressing lncRNA ANRIL was significantly higher than that in cells transfected with pcDNA3.1 (*P* < 0.01, Figure 3A), suggesting the possible involvements of miR-21 in lncRNA ANRIL-associated modulation. In addition, without the induction of H_2_O_2_, cell viability was increased by overexpressing lncRNA ANRIL (*P* < 0.05, Figure 3B). The down-regulation of p53 as well as up-regulation of cyclinD1 and CDK4 were also observed (all *P* < 0.05, Figure 3C, 3D). Moreover, lncRNA ANRIL silencing vector was constructed, leading to down-regulation of lncRNA ANRIL (*P* < 0.001, Figure 3E). Silencing lncRNA ANRIL inhibited miR-21 (*P* < 0.01, Figure 3F), while H_2_O_2_ induction down-regulated the expression of lncRNA ANRIL (*P* < 0.001) and inhibited miR-21 (*P* < 0.01) (Figure 3G), representing the close involvement of miR-21 and lncRNA ANRIL in the regulation of H_2_O_2_ damage.

**Figure 3:** **LncRNA ANRIL could up-regulate miR-21 expression in HLECs.** HLEC SRA01/04 cells were transfected with pcDNA3.1 or pc-ANRIL, and untransfected cells were acted as control. (**A**) and (**E**–**G**) expression of lncRNA ANRIL and miR-21 were determined by RT-qPCR. (**B**) Cell viability was measured by CCK-8 assay. Data are shown as the mean ± SD of three independent experiments. *, *P* < 0.05; **, *P* < 0.01; ***, *P* < 0.001.

### Overexpression of lncRNA ANRIL affected H_2_O_2_-treated HLECs through up-regulating miR-21

Whether dysregulated miR-21 could alter the effects of lncRNA ANRIL on H_2_O_2_-treated HLEC SRA01/04 cells was studied. First of all, the transfection efficiency of miRs was analyzed. In Figure 4A, miR-21 level in cells transfected with miR-21 inhibitor was markedly lower than that in cells transfected with inhibitor-NC (*P* < 0.001), suggesting that miR-21 was silenced successfully after cell transfection. Then, cells co-transfected with pcDNA3.1 (pc-ANRIL) and miR-21 inhibitor (inhibitor-NC) or untransfected cells were treated with H_2_O_2_, and cell injury was evaluated. We found effects of lncRNA ANRIL on cell viability, proliferation and apoptosis were all reversed by miR-21 inhibition, as evidenced by reduced cell viability (*P* < 0.05, Figure 4B), up-regulated p53 as well as down-regulated cyclinD1 and CDK4 (*P* < 0.05 or *P* < 0.01, Figure 4C, 4D), increased apoptotic cells (*P* < 0.05, Figure 4E, 4F), and up-regulated Bax and cleaved caspase-3 as well as down-regulated Bcl-2 (Figure 4G), when compared to the H_2_O_2_ + pc-ANRIL + inhibitor-NC group. The γH2AX staining positive cells were reduced by miR-21 inhibition (*P* < 0.05, Figure 4H). Besides, in order to further verify miR-21 was the miRNA that ANRIL could directly interact with, the miR-34a inhibitor and miR-122-5p inhibitor were synthesized and we transfected them into cells. As shown in Figure 5, miR-34a (*P* < 0.001, Figure 5A) and miR-122-5p (*P* < 0.01, Figure 5C) were separately down-regulated in miR-34a inhibitor- and miR-122-5p inhibitor-transfected HLEC SRA01/04 cells. Besides, miR-34a inhibition or miR-122-5p down-regulation could not affect the beneficial function of pc-ANRIL on cell viability (Figure 5B–5D). Results indicated that lncRNA ANRIL might affect H_2_O_2_-treated HLECs through up-regulating miR-21.

RETRACTED

**Figure 4:** **miR-21 inhibition reversed the effects of lncRNA ANRIL on H_2_O_2_-treated HLECs.** HLEC SRA01/04 cells were transfected with inhibitor-NC or miR-21 inhibitor, and untransfected cells were acted as control. (**A**) Expression of miR-21 was determined by RT-qPCR. Cells co-transfected with pcDNA3.1 (pc-ANRIL) and miR-21 inhibitor (inhibitor-NC) or untransfected cells were treated with 400 μM H_2_O_2_, and non-treated cells were acted as control. (**B**) Cell viability was measured by CCK-8 assay. (**C**, **D**) Expression of p53, cyclinD1 and CDK4 was testified by Western blot analysis. (**E**, **F**) Percentage of apoptotic cells was quantified by flow cytometry assay. (**G**) Expression of proteins related to apoptosis was detected by Western blot analysis. (**H**) γH2AX staining for detection of DNA levels. Data are shown as the mean ± SD of three independent experiments. *, *P* < 0.05; ***, *P* < 0.001.

**Figure 5:** **miR-34a and miR-122-5p could not affect the beneficial effects of LncRNA ANRIL in H2O2-treated HLECs.** HLEC SRA01/04 cells were transfected with inhibitor-NC or miR-34a/miR-122-5p inhibitor, and untransfected cells were acted as control. (**A**) Expression of miR-34a and (**C**) miR-122-5p was determined by RT-qPCR. Cells co-transfected with pcDNA3.1 (pc-ANRIL) and miR-34a/miR-122-5p inhibitor (inhibitor-NC) or untransfected cells were treated with 400 μM H_2_O_2_, and non-treated cells were acted as control. (**B** and **D**) Cell viability was measured by CCK-8 assay. Data are shown as the mean ± SD of three independent experiments. *, *P* < 0.05; **, *P* < 0.01; ***, *P* < 0.001.

### Overexpression of lncRNA ANRIL activated AMPK and β-catenin via up-regulation of miR-21

The involvements of AMPK and β-catenin in lncRNA ANRIL-associated modulation were finally investigated. In Figure 6A, 6B, phosphorylated levels of AMPK were significantly up-regulated by H_2_O_2_ stimulation (*P* < 0.05), and the up-regulation was further increased by lncRNA ANRIL overexpression (*P* < 0.01). In the meantime, phosphorylated levels of AMPK were significantly reduced by miR-21 inhibition relative to the H_2_O_2_ + pc-ANRIL + inhibitor-NC group (*P* < 0.05). The alteration of β-catenin expression after H_2_O_2_ stimulation and ANRIL overexpression with or without miR-21 inhibition was consistent with AMPK phosphorylation (Figure 6C, 6D). The addition of AMPK activator AICAR drove the cellular antioxidant function by promoting production of ROS (*P* < 0.05, Figure 6E). β-catenin activator LiCl promoted cell proliferation by elevating viability (*P* < 0.05, Figure 6F). Most importantly, we then assessed the expressions of ANRIL-miR-21 axis, following utilization of Compound C and XAV939. As expected, block of AMPK or β-catenin induced down-regulation of ANRIL (both *P* < 0.001) and miR-21 (both *P* < 0.001) (Figure 6G), suggesting the significant role of AMPK/β-catenin in ANRIL-miR-21 axis and provided more evidence for the dependency of AMPK and β-catenin in beneficial effects of ANRIL. Above all, results indicated that lncRNA ANRIL could activate AMPK and β-catenin via up-regulation of miR-21. The activation of AMPK and β-catenin promoted the antioxidant function and proliferation of cells.

**Figure 6:** **LncRNA ANRIL activated AMPK and β-catenin in H_2_O_2_-treated HLECs via up-regulation of miR-21.** HLEC SRA01/04 cells co-transfected with pcDNA3.1 (pc-ANRIL) and miR-21 inhibitor (inhibitor-NC) or untransfected cells were treated with 400 μM H_2_O_2_ for 1 h, and non-treated cells were acted as control. Phosphorylation of AMPK (**A**, **B**) and expression of β-catenin (**C**, **D**) were testified by Western blot analysis. (**E**) ROS production was tested through ROS assay; (**F**) cell viability was tested by CCK-8. SRA01/04 cells were transfected with pcDNA3.1 or pc-ANRIL and treated with Compound C or XAV939, and untreated cells were acted as control. (**G**) Expression of lncRNA ANRIL and miR-21 were determined by RT-qPCR. Data are shown as the mean ± SD of three independent experiments. *, *P* < 0.05; **, *P* < 0.01; ***, *P* < 0.001.

RETRACTED

### LncRNA ANRIL and miR-21 were down-regulated in cataract patient tissues

In the *in vivo* experiment, we found that in contrast with normal tissues, lncRNA ANRIL and miR-21 had low expression level in cataract patient tissues (*P* < 0.05 or *P* < 0.01, Figure 7A, 7B). Those data further demonstrated that H_2_O_2_ stimulation caused same results with the *in vivo* assay in which lncRNA ANRIL and miR-21 were down-regulated.

**Figure 7:** **LncRNA ANRIL and miR-21 were down-regulated in cataract patient tissues.** The expression of (**A**) lncRNA ANRIL and (**B**) miR-21 were detected by RT-qPCR. *, *P* < 0.05; **, *P* < 0.01.

### Diagram for our findings

We made abstract diagram for our findings. It suggested in HLEC SRA01/04 cells, H2O2 treatment induced decline of lncRNA ANRIL and miR-21 expression and stimulated HLEC cell damage, regarding proliferation suppression, apoptosis promotion and DNA damage. What’s more, AMPK and β-catenin were involved in the effects of lncRNA ANRIL-miR-21 axis. Besides, *in vivo* experiments showed that expression of lncRNA ANRIL and miR-21 were down-regulated in ARCC, ARNC and ARPC patient tissues compared to the control group.

## DISCUSSION

Currently, surgical intervention and replacement of the cloudy lens are the only treatment for cataract. Hence, the studies focused on the molecular mechanism of cataract should be expanded to explore innovative therapeutic targets. Herein, we constructed oxidative stress model of HLECs and found lncRNA ANRIL could attenuate H_2_O_2_-induced cell injury. miR-21 expression was positively regulated by lncRNA ANRIL expression, and miR-21 inhibition could reverse the effects of lncRNA ANRIL on HLECs under stimulation of H_2_O_2_. Besides, phosphorylation of AMPK and expression of β-catenin were increased by lncRNA ANRIL, possibly through up-regulating miR-21. Block of AMPK and β-catenin led to down-regulation of lncRNA ANRIL as well as miR-21.

Considering that apoptosis of HLECs is the common cellular basis for the formation of non-congenital cataract, whether the oxidative stress model of HLECs was constructed successfully was evaluated according to the alteration of cell proliferation and apoptosis. p53 protein which is kept at low levels in unstressed cells can be stabilized and activated in response to multiple stresses including H_2_O_2_ stimulation, followed by cell cycle arrest and activation of apoptosis pathway [21]. In this study, H_2_O_2_-induced up-regulation of p53 which illustrated H_2_O_2_ might repress proliferation and induce apoptosis. Regulation of the cell cycle, which is driven by cyclins and regulatory partners CDKs, is pivotal for proliferation [22]. CyclinD1 associated with CDK4 can mediate phosphorylation of retinoblastoma protein [23]. In the present study, cell viability and expressions of cyclinD1 and CDK4 were reduced by H_2_O_2_, indicating that H_2_O_2_ repressed HLEC proliferation. Moreover, the H_2_O_2_-induced up-regulation of Bax and down-regulation of Bcl-2 could enhance the release of apoptosis factors, which ultimately led to activation of caspases. Results proved that H_2_O_2_ induced HLEC apoptosis via the intrinsic apoptosis pathway.

RETRACTED

**Figure:** **Abstract diagram. ANRIL, antisense non-coding RNA in the INK4 locus; miR-21, microRNA-21; AMPK, adenosine monophosphate-activated protein kinase.**

Expression of lncRNA ANRIL was dysregulated in HLECs via stable transfection. Then, the effects of lncRNA ANRIL overexpression on H_2_O_2_-treated cells were evaluated. We found lncRNA ANRIL could significantly alleviate H_2_O_2_-induced cell injury via down-regulating p53 and inhibiting intrinsic apoptosis pathway. Effects of lncRNA ANRIL on H_2_O_2_-induced HLECs were consistent with that on cancer cells. Huang et al. have reported that knockdown of lncRNA ANRIL repressed proliferation and induced apoptosis of hepatocellular carcinoma cells (HepG2 and HepG3B) [24]. Previous studies proposed lncRNA ANRIL promoted proliferation of nasopharyngeal carcinoma cells and the expression of p14 which prevented p53 degradation was up-regulated by knockdown of lncRNA ANRIL [25, 26]. Silencing lncRNA ANRIL enhanced apoptosis of bladder cancer cells via up-regulating Bax and cleaved caspase-3 while down-regulating Bcl-2 [27].

miRNAs are small non-coding RNAs of 17-25 nucleotides in length and participate in various biological cellular events. Recently, miRNAs are identified to be involved in cataract development, assisting in investigation of novel diagnostic markers and therapeutic targets [28]. In the meantime, the regulatory mechanism of lncRNA ANRIL is related to miRNA expression. For example, lncRNA ANRIL knocking down repressed proliferation and enhanced apoptosis of human glioma cells via regulation of miR-34a [29]. Proliferation of hepatocellular carcinoma cells was suppressed by lncRNA ANRIL knocking down via regulation of miR-122-5p [30]. Therefore, we focused on the downstream miRNAs to explore the regulatory mechanism of lncRNA ANRIL. miR-21 is an oncomir in many types of tumors, and it can regulate proliferation of bladder cancer cells via regulating p53 [31]. MiR-21 is able to express in various human tissues. Findings have pointed out that miR-21 overexpression could be associated with tissue injuries including inflammation [32]. Wu et al. have proved that HBP1 was not only the target of miR-21 but also the transcriptional activator of p53, indicating the possible involvements of miR-21 in lncRNA ANRIL-associated modulations which was related to p53 [33]. However, whether miR-21 was connected with cataract and function of lncRNA ANRIL was not clear. Hence, in the present study, we measured the expression of miR-21 in HLECs overexpressing lncRNA ANRIL and found the positive correlation between lncRNA ANRIL and miR-21. Furthermore, we also found miR-21 inhibition could effectively abrogate the effects of lncRNA ANRIL overexpression on H_2_O_2_-treated HLECs, verifying that the up-regulation of miR-21 induced by lncRNA ANRIL might be a rational explanation for the protective role of lncRNA ANRIL.

RETRACTED

AMPK is a conserved serine/threonine kinase that intermediates cellular processes including growth, proliferation and survival [34]. β-catenin is a multifunctional protein that acts critical roles in proliferation and apoptosis [35, 36]. Activation of AMPK and β-catenin has been reported to attenuate H_2_O_2_-induced cell injury [37, 38]. Therefore, we finally studied the activity of AMPK and β-catenin. Results showed both AMPK and β-catenin were activated by lncRNA ANRIL and the activation was abated by miR-21 inhibition. Moreover, block of AMPK and β-catenin separately caused by Compound C and XAV939 suppressed the expression of lncRNA ANRIL and miR-21, showing the involvement of AMPK/β-catenin in lncRNA ANRIL-miR-21 axis. Results illustrated that lncRNA ANRIL could activate AMPK and β-catenin via up-regulating miR-21.

In conclusion, we constructed *in vitro* oxidative stress model of HLEC SRA01/04 cells using H_2_O_2_-stimulation. Then, we reported for the first time that lncRNA ANRIL could protect HLECs against H_2_O_2_-induced cell injury via up-regulating miR-21. What’s more, AMPK and β-catenin were activated by lncRNA ANRIL via miR-21. This study laid foundation for the deep investigation of lncRNA ANRIL function in cataract, and provided potential therapeutic targets for treatments of cataract.

## MATERIALS AND METHODS

### Clinical samples

The tissues used in our experiment were explanted from 8 patients with age-related cortical cataract (ARCC), 8 patients with age-related nuclear cataract (ARNC) and 8 patients with age-related posterior subcapsular cataract (ARPC) between March 2017 and March 2018 at The First Affiliated Hospital of Zhengzhou University (Zhengzhou, China). Besides, 6 patients underwent anterior retinal membrane vitrectomy served as control. Inclusion criteria: 24 patients were included according to the Lens Opacities Classification System III (LOCS III), including 8 patients in each ARC classification. Exclusion criteria included high myopia, uveitis, patients with eye trauma or other complicated cataracts of known etiology, glaucoma, myopia, diabetic retinopathy and uveitis as well as other major eye diseases, systemic diseases such as hypertension and diabetes. All procedures were approved by the Ethics Committee.

RETRACTED

### Cell culture and treatment

HLEC SRA01/04 cell line was obtained from the Tumor Center of the Chinese Academy of Medical Sciences (Beijing, China). HLEC SRA01/04 cells were cultured in Dulbecco’s modified Eagle’s medium (DMEM; GIBCO BRL, Grand Island, NY, USA) with 10% fetal bovine serum (FBS; GIBCO BRL) in a humidified incubator filled with an atmosphere consisting of 5% CO_2_ and 95% air at 37°C. For stimulation with H_2_O_2_ (Sigma-Aldrich, St. Louis, MO, USA), cells were incubated in DMEM containing 0, 100, 200, 300-400, 500 and 600 μM H_2_O_2_ for 1 h [39, 40]. Besides, AMPK inhibitor-Compound C (20 μM, for 24 h) and β-catenin inhibitor-XAV939 (1 mM, for 12 h) were separately utilized for cell treatment as indicated.

### Cell transfection

Full-length human lncRNA ANRIL sequences were amplified and ligated into pcDNA3.1 plasmid (Invitrogen, Carlsbad, CA, USA), and the recombined plasmid was referred to as pc-ANRIL. The stable knockdown lncRNA ANRIL vector (si-ANRIL) was generated by the specific target small interference RNA (siRNA). Empty pcDNA3.1 or pc-ANRIL, as well as si-ANRIL were transfected into HLEC SRA01/04 cells with the help of the lipofectamine 3000 reagent (Invitrogen) according to the manufacturer’s instructions. Stable cell line overexpressing lncRNA ANRIL was obtained after selection in culture medium containing 0.5 mg/mL G418 (Sigma-Aldrich) for approximately 4 weeks. MicroRNA (miR)-21 inhibitor, miR-34a inhibitor and miR-122-5p inhibitor as well as its negative control (inhibitor-NC) were synthesized by Shanghai GenePharma Co., Ltd. (Shanghai, China). The lipofectamine 3000 reagent (Invitrogen) was also used for transfection with miR-21 inhibitor or inhibitor-NC. Cells were harvested at 72 h post-transfection in the subsequent experiments.

RETRACTED

### Cell viability assay

A Cell Counting Kit-8 (CCK-8, Dojindo Molecular Technologies, Gaithersburg, MD, USA) was used for measurements of cell viability. In brief, cells (5 × 10^3^ cells/well) were seeded in 96-well plates, and cells were incubated at 37°C for attachment. After treatments, the CCK-8 solution (10 μL/well) was added to the culture medium, and the 96-well plates containing cells were subjected into a humidified incubator at 37°C for 1 h. The absorbance was measured at 450 nm using a Microplate Reader (Bio-Rad, Hercules, CA, USA).

### Apoptosis assay

An FITC Annexin V/Dead Cell Apoptosis Kit with FITC annexin V and PI, for Flow Cytometry (Invitrogen) was used for analysis of apoptotic cells. Briefly, after treatments, cells were collected by Trypsin/EDTA, washed in phosphate buffered saline (PBS), and suspended in binding buffer. Then, cells (5 × 10^5^ cells) were incubated with 5 μL of FITC annexin V and 100 ng of propidium iodide (PI), and the mixture was incubated at room temperature for 15 min. The apoptotic cells were identified and analyzed by using a FACS can (Beckman Coulter, Fullerton, CA, USA). Percentage of apoptotic cells was analyzed by using FlowJo software (Tree Star, San Carlos, CA, USA).

### γH2AX staining

Measurements of DNA damage level were conducted according to the method described in a previous report [41]. Cells probed with fluorescent labelled anti-γH2AX were examined for the values obtaining by flow cytometry.

### TUNEL assay

By means of detection kit-fluorescein (Bio-Rad Laboratories, Hercules, CA, USA) cells death was detected [42]. After culturing and fixing, cells were treated with paraformaldehyde solution (4%) at room temperature, and with Triton X-100 (0.1%) (Bio-Rad Laboratories) on ice. After blocking, TUNEL (Bio-Rad Laboratories) was added to samples and incubated for 1 h in the dark. The percentage of TUNEL-positive cells in was calculated using Mac SCOPE (Bio-Rad Laboratories).

### ROS assay

ROS level was detected by flow cytometry (Beckman Coulter). Cells were prepared in serum-free medium containing 2,7-dichlorofluorescein diacetate (DCFH-DA) (Beijing Biosea Biotechnology, Beijing, China) and reacted for 20 min in the dark. After washing and digesting, cells were collected via centrifugation. The ROS level was detected by flow cytometer (Bio-Rad Laboratories, 488 nm excitation, 521 nm emission).

### Reverse transcription-quantitative PCR (RT-qPCR)

After treatments, total RNA was isolated using Trizol reagent (Invitrogen) according to the manufacturer’s instructions. The expression of lncRNA ANRIL was quantified by using the One Step SYBR^®^ PrimeScript™ PLUS RT-RNA PCR Kit (TaKaRa Biotechnology, Dalian, China) following the suggested protocol. For analysis of miR-21 expression, 500 ng RNA was reversely transcribed to cDNA using the Taqman MicroRNA Reverse Transcription Kit (Applied Biosystems, Foster City, CA, USA). The thermocycling program of reverse transcription was 30 min at 16°C, 30 min at 42°C and 5 min at 85°C. Afterwards, cDNA (50 ng) was acted as template for real-time PCR using the Taqman Universal Master Mix II (Applied Biosystems) according to the manufacturer’s protocol. The thermal cycling conditions were 1 cycle at 95°C for 10 min, followed by 40 cycles of 95°C for 15 s and 60°C for 1 min. GAPDH and U6 were acted as internal control for measurements of lncRNA ANRIL level and miR-21 level, respectively. Relative fold changes were calculated according to the 2^-ΔΔCt^ method [43].

RETRACTED

### Western blot analysis

After treatments, protein of cells was extracted using RIPA buffer (Beyotime Biotechnology, Shanghai, China). Concentration of proteins was quantified using the BCA™ Protein Assay Kit (Pierce, Appleton, WI, USA), and equal amounts of proteins were subjected to SDS-PAGE, followed by transfer to polyvinylidene difluoride (PVDF) membranes. Subsequently, PVDF membranes were blocked at room temperature with 5% bovine serum albumin (BSA) in Tris-buffered saline with 0.5% Tween-20 (TBST). Membranes were incubated at 4°C overnight with primary antibodies specific for p53 (ab131442), cyclinD1 (ab134175), cyclin-dependent kinase 4 (CDK4; ab199728), B cell lymphoma-2 (Bcl-2; ab196495), Bcl-2-associated X protein (Bax; ab182733), pro caspase-3 (ab90437), cleaved caspase-3 (ab49822), AMP-activated protein kinase (AMPK; ab32047), phospho (p)-AMPK (ab131357), β-catenin (ab32572), p14^ARF^ (ab14932), p15^INK4B^ (PA5-49749, Thermo Scientific ®), p15INK4B (PA1-30670) or β-actin (ab8229, all Abcam, Cambridge, UK). Then, PVDF membranes were washed in TBST and incubated with an HRP-conjugated secondary antibody (goat-anti-rabbit, ab205718, Abcam) at room temperature for 2 h. An enhanced chemiluminescence kit (GE Healthcare Bio-Sciences, Pittsburgh, PA, USA) was used for visualization of proteins in those membranes. The intensity of the bands was determined by ImageJ software (National Institutes of Health, Bethesda, MA, USA).

### Statistical analysis

Experiments were performed in triplicate with three repeats. The results were presented as the mean ± standard deviation (SD) using Graphpad Prism 5 software (GraphPad, San Diego, CA, USA). The *P*-values were calculated using unpaired two-tailed *t*-test or multiple *t*-tests. A value of *P* < 0.05 was considered as the threshold for significance.
